RETRACTED

# Effects of miR-124-3p Silencing on Neuronal Damage in the Hippocampus of Depression Rats by Regulating STAT3 Gene

**DOI:** 10.1155/2022/3733656

**Published:** 2022-06-30

**Authors:** Guangping Qin, Zhuo Li

**Affiliations:** ^1^Department of Neurology, Shinan District People's Hospital, Qingdao, Shandong 266100, China; ^2^Second Department of Encephalopathy, Penglai Hospital of Traditional Chinese Medicine, Yantai, Shandong 264000, China

## Abstract

**Objective:**

A large amount of evidence shows that the abnormal expression of miRNA plays an important role in the development of depression. Therefore, we investigated the effect of miR-124-3p on neuronal damage in the hippocampus of depression rats.

**Methods:**

The target genes of miR-124-3p were predicted by the database; the depression model was prepared by subcutaneous injection of corticosterone (CORT), and LV-miR-124-3p asponge lentiviral suspension was given to determine the weight of rats and open-field test, sugar preference experiment, Serum CORT, 5-HT, DA, and NE were measured, observe and record the behavior of rats, including behavior, diet, and hair. The expression of miR-124-3p, STAT3, Bcl-2, and Bax in rat hippocampus was measured. The rat hippocampal neuron cells were extracted and transfected with miR-124-3p inhibitor; the cells were cultured with CORT, and the cell survival rate was evaluated by MTT experiment, and the expressions of miR-124-3p, STAT3, Bcl-2, and Bax in the cells were detected. Luciferase reporter gene verifies the targeted regulation of miR-124-3p on STAT3.

**Results:**

Compared with depression rats, silencing miR-124-3p increased the weight of the rats, increased the number of open-field activities, and significantly improved the general state and pathological state of the rats. The sugar water preference rate was significantly increased, the CORT content in the serum of rats decreased significantly, and the levels of 5-HT, DA, and NE increased significantly. After the treatment of silencing miR-124-3p, the expression level of miR-124-3p was decreased, while the STAT3 mRNA and protein expression levels were increased. And the protein and mRNA expression levels of Bcl-2 were increased, and the Bax protein and mRNA expression were decreased. Cell experiments verified that silencing miR-124-3p increased cell survival, the expression level of miR-124-3p decreased remarkably, while the expression levels of STAT3 mRNA and protein increased significantly. Silencing miR-124-3p reversed the effects of CORT treatment on miR-124-3p and STAT3 in neuronal cells. The luciferase reporter gene experiment confirmed that miR-124-3p targets and regulates STAT3 expression.

RETRACTED

**Conclusion:**

Silencing miR-124-3p may protect hippocampal neurons from damage in depression rats by upregulating STAT3 gene.

## 1. Introduction

Depression is a serious psychiatric disorder associated with cognitive disorder, including physical and psychological symptoms [1, 2]. It is reported that approximately 350 million people worldwide are affected by depression [3], which is a major cause of incapacity to work and imposes a heavy financial and emotional burden on society. The results of a meta-analysis of mental disorders revealed that the risk of suicide in depressed people was 11.2%, much higher than for people with other mental disorders. In contrast, the risk of suicide in other types of mental disorders was 12.7% in total [4]. The overall incidence of depression in the elderly in China was 23.6% [5], and depression was an independent risk factor for death due to various complications (such as heart failure, cancer, and stroke) [6]. Therefore, it is especially vital to further investigate the relevant targets and mechanisms during the development of depression.

Researchers generally believe that an important measure to treat depression is to reduce cognitive disorder [7], and it has been demonstrated that changes in the extracellular matrix in the rat hippocampus can cause cognitive disorder and a chronic depression-like state [8]. Studies show that the occurrence of human depressive symptoms is closely related to hippocampal damage; depression leads to endocrine system disorders in patients, increased levels of cortisol (CORT), and then leads to neurons damage, a key pathological characteristic of patients with depression [9]. Thus, preventing hippocampal neurons from damage is a key direction for depression treatment.

MicroRNAs (miRNAs), as post-transcriptional regulators of gene expression, participate in almost all cellular regulatory processes, and their abnormal expression is closely associated with the pathogenesis of depression [10]. A previous report indicates that miRNAs are of great significance in the pathophysiology of depression and antidepressant drug development [11]. Among the numerous miRNAs, miR-124 is highly expressed in the brain, which is significantly upregulated in depressed rats as well as in postmortem brain and serum samples from depressed patients [12]. Other studies show that miR-124 expression levels are upregulated in the plasma of patients with depression, while their expression levels are decreased after fluoxetine treatment [13]. These studies all suggest that miR-124 may function as a biomarker for diagnosis and response to antidepressant treatment, while studies on whether miR-124-3p protects hippocampal neurons from damage by regulating downstream target expression have not been reported.

RETRACTED

In this study, to further explore the possible effect of miR-124-3p on neurons damage in the hippocampus of depressed rats, we predicted the downstream target gene of miR-124-3p by bioinformatics and further determined whether silencing miR-124-3p protects against neural damage in the hippocampus of rats through target genes.

## 2. Materials and Methods

### 2.1. Materials

Male Sprague-Dawley (SD) rats; CORT purchased from Sigma; rat CORT, 5-HT, DA, and NE kits purchased from Shanghai Zhen Ke Biological Technology Co., Ltd.; LV-miR-124-3p asponge (inhibition vector) and LV-Ctrl (empty vector) synthesized by AtaGenix Laboratories; MTT assay kit purchased from Saint-Bio; dual-luciferase activity assay kit purchased from Shanghai Zeye Biotechnology Co., Ltd.; STAT3, Bcl-2, and Bax antibodies obtained from Cell Signaling Technology; TRIzol reagent purchased from Life Technologies; Bestar™ qPCR RT Kit, SYBR Green qPCR Master Mix, M-MLV reverse transcriptase, and SYBR PreMix Ex Taq GC kit from DBI Bioscience; Lipofectamine 2000 transfection kit from Shanghai Hengfei Biological Technology Co., Ltd.

### 2.2. Methods

#### 2.2.1. Experimental Animals

Thirty male adult SD rats weighing 180-200 g were purchased from Chengdu Dossy Experimental Animals Co., Ltd. [SCXK (Sichuan) 2014-028]. The rats were cultured in a specific pathogen-free environment at 23-25°C and humidity of 35-40%, fed with normal diet and free water. This experiment was approved by the Animal Ethics Committee of our hospital and conformed to the National Institutes of Health guidelines for animal experiments. Animal experiments were conducted in our laboratory animal center, and we tried our best to decrease the suffering of the animals during the experiment.

#### 2.2.2. Bioinformatics Prediction of Target Genes of miR-124-3p

In this study, the target genes of miR-124-3p were predicted with TargetScan (http://www.targetscan.org/vert_72/), miRDB (http://mirdb.org/), and miRTarBase (http://mirtarbase.cuhk.edu.cn/php/index.php), and the intersection of these three databases was used as the final target gene.

#### 2.2.3. Construction of Lentiviral Vector and Cell Transfection

Sequence finding and design of rat MiR-124-3p were done by AtaGenix Laboratories. Recombinant LV-miR-124-3p asponge (suppressor vector) and LV-Ctrl (empty vector) lentiviral expression vectors were synthesized by AtaGenix Laboratories and conformed by sequencing and determined by titer. The prepared recombinant lentiviruses were stored in a -80°C refrigerator for future use.

miRNA-NC and miRNA-124-3p inhibitors were purchased from AtaGenix Laboratories (Wuhan, China). Neonatal rats' hippocampal neurons were seeded in 6-well plates, and when the cells grew to 80% confluence, miR-124-3p inhibitor (50 nM) or miRNA-NC (50 nM) was transfected into neonatal rats' neurons and transfected using Lipofectamine 2000 transfection kit, and after 48 h, collected the cells for the next experiment.

RETRACTED

#### 2.2.4. Establishment of Rat Depression Model and Experimental Grouping [14]

The rats were casually divided into 3 groups, including 10 rats in the blank control group without any treatment. The remaining rats were treated by daily subcutaneous injections of 40 mg/kg corticosterone (CORT) for 21 days continuously to establish a depression model [14]. The rats with successful modeling were casually divided into a depression model group and a miR-124-3p inhibitor group, with 10 rats in each group. Rats in the model group were treated by 10 *μ*L of LV-Ctrl in the rat hippocampus under aseptic conditions; rats in miR-124-3p inhibitor group were treated by 10 *μ*L of LV-miR-124-3p asponge lentivirus suspension (the titer of the virus was 108 TU/mL) in the rat hippocampus under aseptic conditions. Afterwards, the serum and hippocampal tissues of the rats were taken; the behavior of the rats, including movement, diet, and hair, was recorded.

#### 2.2.5. Evaluation of Depression Models

(1) Body weight test: Each mouse was weighed on Day 7, 14, and 21 before and after modeling; (2) open-field test: on the last day of modeling, the horizontal movement of rats was observed by open-field test; (3) sugar preference behavioral test: on the 16th day of CORT injection, the rats were single-housed. Two bottles of sucrose solution (1%, w/v) were placed in each cage for 24 h, and then replace one of them with pure water for 24 h. At the end of the acclimation period, rats were fasted for 24 h. The sucrose preference test was implemented simultaneously each day (9 am), with the rats individually caged and served with bottles containing 100 mL of sucrose solution (1% w/v) and 100 mL of purified water. 24 h later, the volume of sucrose solution and pure water consumed was recorded and the sucrose preference percentage was determined using the following formula. Sugar preference rate% = sugar consumption/(sugar consumption + pure water consumption) x 100%; (4) determination of serum CORT, 5-HT, DA, and NE concentrations: The serum of rats was taken and the contents of CORT, 5-HT, DA, and NE were analyzed by ELISA kits.

#### 2.2.6. HE Staining

Rat hippocampal tissues were fixed by formaldehyde, stained by hematoxylin-eosin (HE), and then determined with light microscopy.

#### 2.2.7. Hippocampal Neurons Collection in Rats [15]

Neonatal rats were used to isolate their brain tissue and remove hippocampal tissue. Rat hippocampal neurons were collected by the method of enzymatic digestion, and single cell suspension was prepared by adding phosphate buffered saline (PBS) to adjust the cell density of hippocampal neurons to 1 x 10^6^ cells/mL.

RETRACTED

#### 2.2.8. CORT-Treated Cells and MTT Assay

Rat hippocampal neurons were transfected by miR-124-3p inhibitor for 24 h and cultured in DMEM medium containing 500 *μ*mol·L^−1^ CORT for another 24 h, after which MTT assay was conducted. The DMEM medium containing CORT was replaced with DMEM medium containing 20 *μ*l MTT solution, and the culture was continued for 4 h at 37°C. Afterwards, 200 *μ*l of dimethyl sulfoxide was supplemented to completely dissolve the formazan crystals. The absorbance of each well was read at 570 nm by a Synergy H1 fully functional microplate reader.

#### 2.2.9. Dual-Luciferase Activity Assay

Using TargetScan (http://www.targetscan.org) to predict the binding site of STAT3 and miR-124-3p, the recombinant reporter plasmids pmir-STAT3 wild-type (wt) -3′UTR and pmir- STAT3 mutant (mut) -3′UTR were constructed: the 3′ UTR of STAT3 was amplified from 293T cell cDNA and cloned into the pmir plasmid to construct the pmir-STAT3 wt-3′ UTR, while the pmir- STAT3 mut-3′ UTR was constructed by Stratagene mutation kit according to the instructions. After 48 hours of cell culture, pmir- STAT3 wt-3′ UTR and pmir- STAT3 mut-3′ UTR were co-transfected with miR-124-3p inhibitor or miR-NC inhibitor with lipofectamine™ 2000. After 48 h, the relative activity of luciferase in each group was measured.

#### 2.2.10. Western Blotting

Rat hippocampal tissue proteins were isolated with lysis buffer for western blot analysis. In brief, 20 *μ*g of protein was solubilized in 10-15% SDS/PAGE and transferred to a polyvinylidene fluoride membrane. The membrane was first blocked for 2 h, and then the membrane was maintained with the primary antibody overnight at 4°C overnight, including STAT3 (1 : 1,000), Bcl-2 (1 : 1,000), Bax (1 : 1,000), and GAPDH (1 : 2,000). Then, the membrane was removed and incubated with horseradish peroxidase-labeled secondary antibody at room temperature, developed with ECL chemiluminescence, recorded with a digital camera, and analyzed using ImageJ software. Results were normalized with GAPDH.

#### 2.2.11. Real-Time Quantitative Fluorescence PCR Assay

Total RNA from rat hippocampal tissue was extracted using TRIzol reagent. RNA concentration was determined by spectrophotometer (1.9 < A260/A280 <2.0). To determine miR-124-3p expression, reverse transcription was carried out using the Bestar™ qPCR RT Kit, miRNA expression was measured on an ABI 7500 qPCR system using SYBR Green qPCR Master Mix, and U6 was recruited as an internal reference. Expression level of mRNA was quantified with M-MLV reverse transcriptase and SYBR PreMix Ex Taq GC kit. All primers were obtained from Invitgen, and GAPDH was employed as an internal reference for mRNA. The relative expression of genes was analyzed with the 2^−*ΔΔ*Ct^ method. The efficiency of the PCR should be between 90 and 110% (3.6 > slope >3.1). All primers were listed as below: miR-124-3p: Forward 5′- GCGCTAAGGCACGCGGTG-3′; Reverse 5′-GTGCAGGGTCCGAGGT-3′; STAT3: Forward 5′-TGGAGAAGGACATCAGCGGT-3′; Reverse 5′-TGGTCTTCAGGTATGGGGCA-3′; U6: Forward 5′- CTCGCTTCGGCAGCACA-3′; Reverse 5′-AACGCTTCACGAATTTGCGT-3′.

RETRACTED

### 2.3. Statistical Analysis

Statistical analysis was conducted by SPSS 21.0 (IBM corporation, Armonk, NY, USA). Values are expressed as mean ± SD. The *t*-test was employed to compare the data of the two groups, and the one-way ANOVA to compare the data of the three groups. *P* < 0.05 was considered significant.

## 3. Results

### 3.1. Analysis of miR-134-3p Target Gene Prediction Results

TargetScan database prediction resulted in 1547 target genes corresponding to miR-134-3p; miRDB database prediction resulted in 683 target genes; miRTarBase database prediction resulted in 9 target genes (Figure 1(a)); and a total of 6 target genes were obtained by intersection of the three databases. We selected the target gene of interest, STAT3, for our study (Figure 1(b)).

### 3.2. Comparison of General Status in Depressed Rats

The depression model rats had decreased body weight and decreased number of open-field activities compared with the blank control group. And after silencing miR-124-3p, the rats had increased body weight and increased number of open-field activities (Figure 2, Table 1); the observation results of the behavioral parameters of the rats show that the rats in the blank control group were energetic, had normal diet, and had bright hair; the rats in the model group were apathetic, had no diet, and had dim hair; the rats in the miR-124-3p inhibitor group were slightly apathetic, had no diet, and the hair was slightly dim. From Table 2, it can be seen that the sugar preference in the model control group was evidently reduced compared with the normal control group, while enhanced compared with the model control group. The CORT content in the serum of rats from the model group was significantly increased compared with the normal control group. And the levels of 5-HT, DA, and NE were significantly decreased, and the content of CORT in the serum of the rats from the miR-124-3p inhibitor group could be pronouncedly decreased, and the levels of 5-HT, DA, and NE were significantly increased (Figure 3).

RETRACTED

### 3.3. HE Staining Results of Rat Hippocampus

The results of HE staining show that hippocampus cells of control rats were neatly arranged and tight, the nucleoli of the cells were clearly visible, and the chromatin was evenly arranged. In the model group, the cells were disorganized and were loosely arranged, the pyramidal cell layer was thin, and the cell edge was blurred. The above results suggested that the depression model of rats was successfully built. Compared with rats in the model group, the cells of rats in the miR-124-3p inhibitor group were more closely arranged, the cell density was slightly greater, and the pyramidal cell layer was thick indicating that silencing miR-124-3p was able to reduce CORT-induced hippocampal damage (Figure 4).

### 3.4. Expression of MiR-124-3p, STAT3, Bcl-2, and Bax in Hippocampal Tissues

The expression of miR-124-3p was evidently higher, the mRNA and protein expression levels of STAT3 were pronouncedly decreased, the protein and mRNA expression levels of the inhibitor of apoptosis Bcl-2 were downregulated, and the protein and mRNA expression levels of the apoptosis-promoting factor Bax were enhanced in the hippocampal tissues of the model group than that of the blank control group. Compared with the model group, the expression levels of miR-124-3p were decreased, the mRNA and protein levels of STAT3 were increased, the Bcl-2 protein and mRNA expression levels were increased, and the Bax protein and mRNA expression were decreased in the hippocampal tissues of the miR-124-3p inhibitor group (Figures 5 and 6).

### 3.5. Effect of the Silencing miR-124-3p on the Cell Viability of Neonatal Rat Hippocampal Neurons

MTT assay results show that the viability of hippocampal neurons in neonatal rats was evidently decreased after treatment with CORT; however, silencing miR-124-3p reversed the results induced by treatment with CORT and promoted the enhanced viability of hippocampal neurons (Figure 7).

### 3.6. Effect of Silencing miR-124-3p on STAT3, Bcl-2, and Bax in Neonatal Rat Hippocampal Neurons

After CORT treatment of neonatal rat hippocampal neurons, the expression level of miR-124-3p was evidently increased, while the STAT3 protein and mRNA levels were pronouncedly downregulated, the protein and mRNA expression levels of the inhibitor of apoptosis Bcl-2 were decreased, and the protein and mRNA expression levels of the apoptosis-promoting factor Bax were upregulated. After the treatment of silencing miR-124-3p, the expression level of miR-124-3p was decreased, while the STAT3 mRNA and protein expression levels were increased. And the protein and mRNA expression levels of Bcl-2 were increased, and the Bax protein and mRNA expression were decreased (Figures 8 and 9). Silencing miR-124-3p reversed the effects of CORT treatment on miR-124-3p and STAT3 in neurons.

RETRACTED

### 3.7. MiR-124-3p Targeting STAT3

MiR-124-3p has a potential paired sequence region with the STAT3 3′ -UTR region. The results of luciferase reporter gene show that the activity of dual-luciferase was significantly decreased in STAT3-3′UTR-Wt + miR-124-3p compared with the STAT3-3′UTR-Wt + NC group; the difference in dual-luciferase activity was not statistically significant in the STAT3-3′UTR-Mut + miR-124-3p STAT3-3′UTR-Mut + NC group, indicating that miR-124-3p bond with STAT3 (Figure 10).

## 4. Discussion

Depression is a serious mental illness, which seriously influences the physical and mental health of patients and poses burden on patients' families. Currently, the method used to treat depression is not ideal. Although clinical drug therapy replaces electroconvulsive therapy, long-term use of drugs will have toxic and side effects on the body, so the way of drug therapy is still not an ideal method. Therefore, from the pathogenesis of depression as a starting point, finding novel targets for the treatment of depression is vital. At present, due to the development of bioinformatics, it provides a more convenient method for the search of target genes for disease treatment, which has a very far-reaching significance for the treatment of diseases. Clinically, it is believed that the main pathological feature of depression is endocrine dysregulation, which in turn leads to increased levels of CORT, which can induce neurons damage in the hippocampus [16]. Therefore, protecting hippocampal neurons from damage is a novel direction for depression treatment. Here, the protective effect of silencing miR-124-3p was found to regulate STAT3 gene on neuronal damage in the hippocampus of CORT-induced depressive rats.

A previous study shows that miR-124 is a miRNA closely related to depression. For example, it was pointed out that due to the separation of pups from mothers, mothers suffer from depression which in turn leads to the upregulation of some miRNAs, which also include miR-124 [17]. MiR-124 also targets the glucocorticoid receptor (GR), and activation of GR inhibits miR-132, which in turn reduced BDNF expression, which is closely related to depression. MiR-124 is also a neural-specific miRNA and involved in neuronal differentiation. Overexpressing miR-124 in neuroprogenitor, embryonic stem cells, and glioma cells has been shown to lead to forced differentiation of neurons [18]; *in vivo* experimental results demonstrate that miR-124 is able to advance neurogenesis during in development of the brain [19]. A study demonstrated that miR-124-3p, an essential miR for neuronal identity, is highly abundant in neuronal exosomes [20]. In summary, miR-124 is an important regulator of hippocampal neurogenesis. Therefore, the protective effect of silencing miR-124-3p on CORT-induced hippocampal neurons damage at the animal and cellular levels was explored. The results reveal that miR-124-3p was evidently upregulated in the hippocampal tissue of depressed rats, and the general symptoms of depressed rats were significantly improved after silencing miR-124-3p, and the pathological damage was also significantly improved. Next, we isolated neonatal rat hippocampal neurons and silenced miR-124-3p, and it was found that silencing of miR-124-3p reversed CORT-induced damage and increased neurons viability, along with upregulated expression of the apoptosis-inhibiting protein Bcl-2 and inhibited expression of the apoptosis-promoting protein Bax. The above results all indicate that silencing miR-124-3p can protect hippocampal neuronal damage induced by CORT, which in turn plays a key role in reducing depressive damage.

RETRACTED

Additionally, the downstream target genes of miR-124-3p were predicted by bioinformatics and finally selected STAT3 as the downstream target gene of miR-124-3p for study. STAT3 was identified as an important factor in emotional responses, related to depression, schizophrenia, and bipolar disorder, and found to be a key coordinator of cytokine activation in cellular immune responses, and in the “immune hypothesis,” it has a close link to psychopathology [21–23]. In addition to cytokines, the activation of STAT3 can also reflect the role of upstream regulators related to neurological function, including growth factors, hormones, and endocannabinoids [24, 25]. Kwon et al. revealed that STAT3 regulates depression-related behaviors via neuronal M-CSF-mediated synaptic activity [26]. In view of the above reports, targeting STAT3 has the potential to be an important approach for the treatment of depression; we found that silencing miR-124-3p promoted the expression of STAT3 in neuronal CORT damage experiments, and dual-luciferase experiments confirmed that miR-124-3p and STAT3 have targeted regulation.

To conclude, silencing miR-124-3p improves CORT-induced hippocampal neuronal damage in depression, and silencing miR-124-3p may function protectively by targeting STAT3, which offers a new perspective for depression treatment.

## Figures and Tables

**Figure 1:** Prediction results of miR-134-3p target gene.

**Figure 2:** Weight change of rats.

**Figure 3:** Expression levels of CORT, 5-HT, DA, and NE in rat serum. #*P* < 0.05, compared with the control group; ∗*P* < 0.05, compared with the model group.

RETRACTED

**Figure 4:** Results of HE staining.

**Figure 5:** Protein expression of STAT3, Bcl-2, and Bax in hippocampus. #*P* < 0.05, compared with the control group; ∗*P* < 0.05, compared with the model group.

**Figure 6:** MRNA expression levels of miR-124-3p, STAT3, Bcl-2, and Bax in hippocampus. #*P* < 0.05, compared with the control group; ∗*P* < 0.05, compared with the model group.

**Figure 7:** The result of cell viability test. #*P* < 0.05, compared with the control group; ∗*P* < 0.05, compared with the model group.

**Figure 8:** The expression levels of STAT3, Bcl-2, and Bax protein in hippocampal neuron cells. #*P* < 0.05, compared with the control group; ∗*P* < 0.05, compared with the model group.

**Figure 9:** mRNA expression levels of miR-124-3p, STAT3, Bcl-2, and Bax in hippocampal neuronal cells. #*P* < 0.05, compared with the control group; ∗*P* < 0.05, compared with the model group.

**Figure 10:** Luciferase reporter experiment verifies the targeting relationship between miR-124-3p and STAT3. #*P* < 0.05, compared with the control group; ∗*P* < 0.05, compared with the mRNA-NC group.

**Table 1:** Results of the number of open-field experimental activities.

	Control	Model	miR-124-3p inhibitor
Contact time (S)	42.18 ± 3.56	64.54 ± 4.31^#^	53.45 ± 3.21 ∗
Number of crossings (times)	94.87 ± 4.21	129.6 ± 4.97^#^	117.3 ± 4.58 ∗
Number of rearing (times)	17.49 ± 3.89	24.61 ± 3.99^#^	21.11 ± 2.11 ∗

**Table 2:** Effect of silencing miR-134-3p on glucose preference in rat model of depression induced by CORT.

	Sugar preference/(%)
Control	94.87 ± 4.21
Model	43.8 ± 5.8 ^#^
miR-124-3p inhibitor	83 ± 8.9 ∗

## Data Availability

The labeled dataset used to support the findings of this study is available from the corresponding author upon request.
